The article "Impact of the Built Environment on Residents' Health: Evidence from the China Labor Dynamics Survey in 2016" was published in 2023. Journal: J Environ Public Health.

# Impact of the Built Environment on Residents' Health: Evidence from the China Labor Dynamics Survey in 2016

**DOI:** 10.1155/2023/3414849

**Published:** 2023-02-01

**Authors:** Feng Lan, Jingyu Pan, Yulin Zhou, Xin Huang

**Affiliations:** ^1^School of Management, Xi'an University of Architecture and Technology, Xi'an 710055, China; ^2^Key Research Base of Philosophy and Social Sciences In Shaanxi Universities-Research Center of Green Development and Mechanism Innovation of Real Estate Industry in Shaanxi Province, Xi'an, China

## Abstract

In the process of China's rapid urbanization, the health level of residents has been improved to a great extent. However, with the expansion of urban scale and spatial restructuring, a series of urban environmental problems have posed new challenges to public health. However, the impact of the built environment on residents' health is controversial, and the applicability of the conclusions based on western urban sprawl in China is not clear enough. In addition, the exploration of the impact path of the built environment on health is still not comprehensive and in-depth. Based on the China Labor Dynamics Survey (CLDS) in 2016 and relevant statistical yearbook data, this study explored the impact of the built environment at community and urban scale on residents' health and its age heterogeneity and further explored the mediating role of physical exercise, neighborhood support, and community safety. According to the research, the urban and community-built environment has significant impacts on residents' health, and the impact is significantly different at different scales. In addition, there is a significant difference in the impact of built environment factors on residents' health among populations with different life cycles. From the perspective of the impact path, greening coverage can improve residents' self-rated health by enhancing the perceived safety of living in the community. In contrast, the high community population density will not only weaken the degree of neighborhood support but also reduce the perception level of community residential safety, thus damaging residents' health. In short, from the perspective of environmental intervention, the previously mentioned results put forward possible suggestions on strengthening the construction of a healthy living environment so as to maximize the health effectiveness of cities and communities.

## 1. Introduction

As the first medium and long-term health plan in China, the outline of the Healthy China 2030 Plan proposes to take the construction of healthy cities and towns as an important starting point for the construction of a healthy China and to promote the coordinated development of cities and people's health. In the past high-speed and fast-paced urbanization process, the construction of medical and health infrastructure has been constantly promoted, providing convenient and affordable medical security for residents and achieving significant improvement in the health level of the group. However, the massive influx of population and the disorderly expansion of urban space have also brought about the imbalance of employment, education, entertainment, and living space, resulting in the continuous increase of the proportion of motorized travel. On the one hand, high-frequency motorized travel is easy to cause urban congestion, noise pollution, and traffic safety problems. On the other hand, motorized travel increases the sedentary time of individuals, reduces the frequency and intensity of physical activity, and increases the incidence of chronic diseases. In addition, the noisy and crowded environment is not only harmful to physical health, but it also affects residents' life satisfaction, which in turn has a negative impact on mental health. Therefore, it has become the focus of current research to build a healthy living environment through environmental intervention, improve public health facilities from the supply side, and give full play to community health efficiency.

The article "Impact of the Built Environment on Residents' Health: Evidence from the China Labor Dynamics Survey in 2016" was published in 2023. Journal: J Environ Public Health.

## 2. Literature Review

The built environment at different scales has an impact on residents' health in different ways. According to the existing studies, the impact of the built environment on residents' health is divided into three scales: macro (countries around the world/region), meso (city/county), and micro (street/community) [1]. Built environment factors mainly include density, land use mixture, design, distance to bus stations, and destination accessibility [2, 3]. Many studies based on Western low-density cities have found that with the increase in density, residents' health can be significantly improved. This is because compact cities make the layout of different functional facilities closer, compress the travel distance, and have good street connectivity, which can effectively promote nonmotorized travel, such as the walking and cycling mode [4, 5]. As a result, it can increase their physical activities [6], reduce the risk of obesity, and improve their health. However, the research based on China's national conditions indicated that excessively high-density land use is detrimental to residents' health [7], and high population density will cause a rapid decline in residents' health and comfort [8]. Different from the urban sprawl in western countries, which is mainly characterized by rapid suburban development and decline of central urban areas, China's urban sprawl has not seen a significant decline in the population of inner cities, and the central urban areas are still thriving [9]. At the same time, the urban spatial structure in China is more compact than that of American cities, and the population density is about 5–7 times that of American cities [10]. While excessive urban density often leads to local environmental deterioration and reduction of urban operational efficiency, including weakened neighborhood harmony, crowded public spaces, reduced green coverage ratios, lack of privacy, and increased pressure [11].

The article "Impact of the Built Environment on Residents' Health: Evidence from the China Labor Dynamics Survey in 2016" was published in 2023. Journal: J Environ Public Health.

In addition to density and diversity, scholars have found that some urban and community design factors are also related to residents' health, such as green open spaces. At the same time, the research at the urban scale will also focus on road traffic organization. A good slow traffic network can provide a safe walking environment for residents [12], which is conducive to improving residents' willingness to walk and use bicycles [13]. Among all kinds of travel modes, walking has the highest health effect, followed by bus and subway, and private cars are the lowest and far lower than the walking and public transportation [14]. Outdoor activity spaces such as parks are distributed in walkable living circles near the community which can significantly stimulate the residents' willingness to engage in physical activities [15] and help reduce obesity and overweight [16, 17]. In addition, green spaces can reduce the risk of cardiovascular and respiratory diseases by improving urban air quality [18] and can also relieve mental stress [19]. In general, there is no clear and unified answer to the relationship between the built environment factors and residents' health in the existing literature.

Based on the literature review, some aspects in this study are worthy of further research. First, most previous studies only focused on the community-built environment, and only a very limited number of studies have considered the built environment factors both at the community scale and urban scale [20]. Considering the diversity of residents' daily travel modes and the exposure to activities that may extend far beyond the community, it is reasonable to assume that residents' health will be affected by the built environment at different scales simultaneously. Therefore, it is necessary to take both the community and urban scales into consideration. Second, some studies believe that the relationship between the built environment and residents' health is affected by other factors, but there are few studies on the impact mechanism of the built environment on residents' health, and most of them are conducted from the perspective of health behavior. Thus, three mediating variables, namely, physical exercise, neighborhood support, and community safety, were included in this study to explore health behavior and its extrinsic pathways. Finally, the health evaluation dimensions selected in the existing relevant research are insufficient, focusing on physiological health and adopting objective indicators such as BMI and waist-hip ratio. The gap in subjective health research needs to be filled.

The article "Impact of the Built Environment on Residents' Health: Evidence from the China Labor Dynamics Survey in 2016" was published in 2023. Journal: J Environ Public Health.

The remainder of this study is structured as follows: in Section 2, we introduced data sources, descriptive statistics, and model building. The empirical analysis was reported in detail in Section 3. In Section 4, we further discussed the research results and provided corresponding implications.

## 3. Materials and Methods

### 3.1. Data Sources

There are two sources of data used in this study. One is the China Labor Force Dynamic Survey (CLDS) data used to obtain individual household attributes and community-built environment data. The second data source is the Statistical Yearbook of Chinese Cities and the Statistical Yearbook of Urban and Rural Construction used to obtain urban-built environment data.

CLDS is a comprehensive survey project carried out by the Social Science Survey Center of Sun Yat sen University. The survey adopts a multistage stratified probability proportionate to labor size (PPS) sampling method, covering social, economic, demographic, environmental, and other aspects from individuals to families to communities. The project has conducted a follow-up survey every two years since 2012 so as to learn about the change trend of social labor force, families, and communities across China. The survey sample taken by CLDS is very representative nationwide, and it includes labor force aged 15–64 from 29 provinces and cities outside Hong Kong, Macao, Taiwan, Tibet, and Hainan. Based on its large sample base, wide survey area, and high representativeness, it is suitable for systematic statistical research and can provide true and reliable data.

At present, CLDS has released the data of 2012, 2014, and 2016 to the society, and this study uses the data of CLDS 2016. Due to the large difference between urban and rural built environments in China, urban samples were taken into account in this study. Finally, 4,641 valid samples were selected from 130 communities in 55 cities in China after removing the samples that the participants did not know the answer or refused to answer the question as well as the samples which did not meet the analytical conditions.

### 3.2. Variable Definition and Description

#### 3.2.1. Explained Variable

The explained variable in this study is residents' health. Health indicators can be roughly divided into objective and subjective indicators. Compared with objective health, self-rated health is simpler, but it is an assessment made by individuals based on their own perception and actual physiological and psychological state and has been proved to be highly correlated with the prediction of mortality and disability rates [21, 22]. At present, this indicator was widely used in residents' health research, and this study also adopted self-rated health as the measurement of individual health. Individual health variables were measured by the question “How do you think your current health is?” The answers included “very healthy,” “healthy,” “ordinary,” “relatively unhealthy,” and “very unhealthy,” and the assigned values are 1, 2, 3, 4, and 5, respectively. In this study, the original assignment order is reversely adjusted, and the higher changed score indicates a better self-rated health status.

The article "Impact of the Built Environment on Residents' Health: Evidence from the China Labor Dynamics Survey in 2016" was published in 2023. Journal: J Environ Public Health.

#### 3.2.2. Explanatory Variable

The core explanatory variables of this study are built environment characteristics, which will be measured at both community and urban spatial scales. Based on the availability of data from CLDS2016, this study focuses on the density, diversity, and design of the built environment factors at the community scale. The “density” was measured by community population density, and the categorical density was adopted to explore the nonlinear impact of community density on residents' health [23]. The “design” was measured by green coverage ratio. At the same time, considering that environmental pollution has a great impact on residents' health, it is also included in the design dimension for regression analysis. The environmental pollution was calculated by the weighted average of air pollution, water pollution, soil pollution, and noise pollution in the community questionnaire. The “diversity” was reflected by the provision of public infrastructure and service facilities closely related to the daily life of residents in the community, mainly including whether there are primary schools, junior high schools, sports venues/fitness centers, activity rooms for the elderly, libraries, squares/parks, playgrounds, and hospitals/private clinics. If there are such facilities, the value will be 1; if there are no such facilities, the value will be 0. Finally, the diversity score will be obtained by summing them up.

The built environment variables at the urban scale include population density reflecting “density” in urban municipal districts, the road area ratio and green area ratio reflecting “design” in urban municipal districts, buses per 10,000 people and rail transit reflecting “public transport accessibility,” and land use mixture reflecting “diversity.” Besides, in order to control the difference in the built environment among different urban scales, the variable of urban population size was added in this study.

The article "Impact of the Built Environment on Residents' Health: Evidence from the China Labor Dynamics Survey in 2016" was published in 2023. Journal: J Environ Public Health.

#### 3.2.3. Control Variables

Referring to prior studies, this study selected the socio-economic characteristics of individuals and households as well as individual behavioral variables, and the data come from CLDS2016. Specifically, the control variables include gender, age, marital status, educational level, health insurance, household income per capita, car and motorcycle ownership, and history of smoking and alcohol intake. Considering that previous studies have found a U-shaped relationship between age and residents' health, the squared term of age was included in this study.

#### 3.2.4. Mediating Variables

In the mechanism test of the built environment on residents' health, variables of the physical exercise, neighborhood support, and community safety will also be involved. The exercise frequency and intensity of the participants were comprehensively taken into consideration in the physical exercise variable. We assigned a value of 3 to the participants who exercised 3 times per week or more and the sessions last for more than 30 minutes, a value of 1 to those who had no exercise per week, and a value of 2 to others. Neighborhood support was measured by the questionnaire “Do you provide mutual assistance with your neighbors in your community (village)?” The options of “very unfamiliar,” “not very familiar,” “ordinary,” “relatively familiar,” and “very familiar” were assigned with the value from 1 to 5 successively. The community safety variable was also conducted in an ordered category by the question “How do you think of your community safety?” The options of “very unsafe,” “not very safe,” “relatively safe,” and “very safe” were assigned with values from 1 to 4 in sequence. The larger the value is, the safer it is. The descriptive statistical analysis of variables selected in this study is shown in Table 1.

### 3.3. Model Construction

In this study, the individual, household, community, and urban levels were involved simultaneously, which means that individuals from the same spatial unit were affected by the same environmental factors and the health level of residents was also spatially correlated. Theoretically, the research data with a nested structure violated the assumption of multiple regression on sample independence. To solve the problem of data nesting, a multilevel model or clustered robust standard errors were usually employed for regression analysis [24, 25]. In this study, we attempted to adopt a multilevel model, but the null model test shows that the intraclass correlation coefficient (ICC) of residents' self-rated health is 2% at the urban scale and 5.9% at the community scale, both of which are less than 7%, indicating that the intergroup correlation is low [26]. In other words, the issue of individual spatial dependence in our sample data has no effect on the estimation of the built environment on residents' health at the urban and community scales. The self-rated health (the explained variable) in this study is a set of discrete ordinal variables with the assigned value from 1 to 5, which are suitable for the ranking model. Therefore, the ordered probit model was used to analyze the impact of the built environment on residents' health at the urban and community scales. Although the null model test of the multilevel model shows that the samples have good independence, in order to improve the reliability of the results, this study chose to apply the clustered robust standard errors at the community scale into the regression model to solve the problem of spatial correlation. The basic form of the model is as follows:

(1) $$\begin{array}{c} {\text{Health}}_{i}=\alpha +\beta_{1}BE_{\text{city},i}+\beta_{2}BE_{\text{neighborhood},i}+\beta_{3}SE_{i}+\varepsilon \text{.} \end{array}$$

In this equation, Health_*i*_ represents the individual's self-rated health level, *BE*_city,*i*_ represents the built environment variable matrix at the urban scale, *BE*_neighborhood,*i*_ refers to the built environment variable matrix at the community scale, *SE*_*i*_ is the socio-economic attribute variable matrix of individuals and households, *β*_1_ and *β*_2_, respectively, are the influence coefficients of built environment factors on the individual health level at the urban and community level, *β*_3_ represents the influence coefficient of the socio-economic attribute at the individual and household level on residents' health, and *ε* represents the error terms.

The article "Impact of the Built Environment on Residents' Health: Evidence from the China Labor Dynamics Survey in 2016" was published in 2023. Journal: J Environ Public Health.

In the context of Chinese culture, considering that the built environment has a weak causal relationship with residents' unhealthy behaviors such as smoking and drinking, but it may be closely related to residents' health status, therefore, in reference to the model setting of previous studies [27], this study included the unhealthy behaviors such as the history of smoking and alcohol intake as exogenous variables in the model. Given that groups who own cars and motorcycles will give priority to nonmotorized travel, therefore, the condition of owning cars and motorcycles was also included in the model as control variables to reduce estimation errors caused by omitted variables and improve the reliability of regression results. After incorporating individual behaviors, the model is set as follows:

(2) $$\begin{array}{c} {\text{Health}}_{i}=\alpha +\beta_{1}BE_{city,i}+\beta_{2}BE_{\text{neighborhood},i}+\beta_{3}SE_{i}+\beta_{4}\text{Behaviors}+\varepsilon \text{.} \end{array}$$

In this equation, Behaviors represents the behavioral variable matrix of whether an individual smokes, drinks, and whether a family owns a car or motorcycle, *β*_4_ represents the influence coefficient of the individual and family behavior variables on residents' health, and *ε* represents the error terms.

The built environment can not only directly affect the health of residents but can also be affected by other factors. At present, there are few empirical studies on the impact mechanism of the built environment on residents' health, and most of them are analyzed from the perspective of physical activity, lacking research on social capital and the environmental exposure path. In this regard, this study not only considers the path of health behavior but also incorporates the path of the social environment, mainly involving three intermediary variables: physical exercise, neighborhood mutual aid, and community perceived safety. In this study, the stepwise regression method was used to analyze the relationship between the community-built environment, the mediating variables, and residents' health. The bootstrap method was used to test the significance of the mediating effect. The model used in this part of the empirical analysis is as follows:

(3) $$\begin{array}{c} {\text{Health}}_{i}=\alpha +\beta_{1}BE_{\text{neighborhood},i}+\beta_{2}SE_{i}+\beta_{3}\text{Behaviors}+\varepsilon \text{,} \end{array}$$

(4) $$\begin{array}{c} M_{i}=\beta_{0}+\beta_{1}BE_{\text{neighborhood},i}+\beta_{2}SE_{i}+\beta_{3}\text{Behaviors}+\varepsilon_{i}\text{,} \end{array}$$

(5) $$\begin{array}{c} {\text{Health}}_{i}=\beta_{0}+\beta_{1}BE_{\text{neighborhood},i}+\delta M_{i}+\beta_{2}SE_{i}+\beta_{3}\text{Behaviors}+\varepsilon_{i}\text{.} \end{array}$$

In this equation, Health_*i*_ represents the individual's self-rated health level; *BE*_neighborhood,*i*_ refers to the built environment variable matrix at the community scale; *SE*_i_ is the socio-economic attribute variable matrix of individuals and households; Behaviors represents the behavioral variable matrix of whether an individual smokes, drinks, and whether a family owns a car or motorcycle; *M*_*i*_ represents the intermediary variable of physical exercise, neighborhood mutual aid, and community security.

## 4. Results

Models 1 to 4 in Table 2 show the estimated results of the total effects of the built environment on residents' health at different scales. After controlling the socio-economic attributes of individuals and households, in Model 1, we only considered the impact of the built environment on residents' health at the urban level. In Model 2, we only estimated the impact of the built environment on residents' health at the community level. The built environment variables of Model 1 at the urban scale and Model 2 at the community scale were combined into Model 3, and regression analysis is carried out by using formula (1). On this basis, the individual behavioral variables were incorporated into Model 4 as the benchmark model, and formula (4) is used to explore the impact of the built environment on residents' health at the urban and community scales. The estimated results show that the built environment at both urban and community scales is correlated with residents' health, which indicates that there is a hierarchical relationship between the built environment and residents' health. Therefore, it is necessary to consider the characteristics of the built environment at both urban and community levels so as to reduce the deviation caused by omitted variables and better analyze the impact of the built environment on the residents' health.

The article "Impact of the Built Environment on Residents' Health: Evidence from the China Labor Dynamics Survey in 2016" was published in 2023. Journal: J Environ Public Health.

### 4.1. Impacts of the Urban and Community Built Environment on Residents' Health

#### 4.1.1. Impacts of the Built Environment on Residents' Health at the Urban Scales

In terms of the characteristics of the built environment at the urban scale, the urban population density is significantly positively correlated with residents' health, that is, the growing urban population density is accompanied by residents' constantly improved self-perceived health status. Regarding the reason, on the one hand, the growing population density slows down the speed of urban sprawl and compacting cities compress the distance to their destinations, thereby improving the convenience of life. As a result, this creates conditions for reducing the use of private cars and promoting nonmotorized modes of travel such as walking and cycling [28, 29], thus reducing the risk of obesity and chronic diseases and improving health by increasing the frequency and intensity of physical activities. On the other hand, a high population density represents a city's higher operating capacity and more effective urban functions [30], which means a stronger carrying capacity of public services, richer medical resources, a more perfect medical insurance system, and also a better medical treatment environment. All of these will play a positive role in promoting residents' health.

There is a significant positive correlation between the road area ratio and residents' health. The main reason is that increasing the supply of road infrastructure can effectively alleviate the urban traffic congestion [31], thus shortening residents' commuting time. Furthermore, a series of problems such as reduced life satisfaction, less sleeping time, physical discomfort, and negative emotions caused by long-distance commuting are alleviated, thereby improving residents' perception of their own health status.

The article "Impact of the Built Environment on Residents' Health: Evidence from the China Labor Dynamics Survey in 2016" was published in 2023. Journal: J Environ Public Health.

Adequate green space ratio has a positive effect on residents' health, which can be attributed to the long-term regulatory effect of green space on the urban environment. In a word, urban green space can alleviate exposure hazards, reduce urban air pollution, and improve residents' physical and mental health [32]. In the urban built environment, bus accessibility, land use mixture, and rail transit accessibility have no significant influence on residents' self-perceived health.

#### 4.1.2. Impacts of the Built Environment on Residents' Health at the Community Scales

Among the built environment factors at the community scale, the population density and green coverage ratio have a significant influence. Community population density has a nonlinear effect on residents' health. When the population density is between 5,000 and 10,000 people per square kilometer, it has a negative impact on residents' health. When exceeding 15,000 people per square kilometer, the population density still has a significantly negative correlation with residents' health, indicating that an extremely high community population density will reduce the residents' health level. This conclusion is different from that of western developed countries. In terms of the experience of western countries with low density in the context of urban sprawl, population density at the community level can help reduce overweight and obesity and is positively correlated with residents' physiological health [33, 34]. However, the results of this study are consistent with the conclusions in the context of high density in China [35]. The possible reason lies in the high population density of communities in China. Excessive population density will lead to a portion of problems such as space congestion, lack of public facilities, environmental pollution, and invasion of private space, which will aggravate the occurrence of obesity and mental diseases and have a negative impact on residents' health.

Among other built environment factors at the community scale, the green coverage ratio also has a positive effect on residents' health, that is, residents living in communities with a higher green coverage ratio have a stronger self-perceived health status. Communities with higher greenness can provide residents with more green space and important places for daily physical exercise, thus enhancing residents' physical activities, relieving mental stress, and improving their mental health and cognitive function [36, 37]. Additionally, a higher greenness level in residential communities can improve the satisfaction and happiness of residents and relieve their psychological stress, promoting their physical and mental health. However, there is no significant correlation between community diversity and residents' health. The possible reason is that although the higher diversity shortened the distance to the destination and promoted nonmotorized travel, there was a limited positive impact of physical activities generated by nonmotorized travel on residents' health. Besides, higher community diversity means more noisy and crowded living conditions, which has a negative impact on residents' health. The positive and negative effects of community diversity interact with each other, resulting in the insignificant impact of community diversity on residents' health.

The article "Impact of the Built Environment on Residents' Health: Evidence from the China Labor Dynamics Survey in 2016" was published in 2023. Journal: J Environ Public Health.

#### 4.1.3. Impacts of Individual and Household Attributes on Residents' Health

Model 4 shows the overall effects of socio-economic attributes of individuals and households and individual behavior on residents' health. Among the individual characteristics, marital status has a significant positive impact on residents' health. The result means that residents who have a happy marriage will have a higher self-perceived health level, which is consistent with Brockmann's conclusion [38]. The residents' educational level is significantly correlated with their health, that is, people with a higher educational level have higher health status, which is consistent with the research conclusion drawn by Lingguo et al. [39]. Individual age has a significant negative impact on residents' self-rated health, and the age square variable has a significant positive correlation with the health level. The result means that there is a “U”-shaped relationship between individual age and health, that is, individual self-perceived health shows a trend from decreasing to increasing mode with the increase of age. This may be because middle-aged people spend more time working and taking care of their families, which leads to insufficient time for exercise on the one hand, and high psychological pressure on the other hand, thus reducing their physical and mental health. Among the variables of household characteristics, the household income per capita shows a consistent impact relationship as expected, that is, the higher the household income per capita, the higher the health level of the residents. In terms of individual behavior, car ownership has a negative impact on residents' health, as the households owing cars have a stronger desire to travel by motorization, which increases the sedentary time and increases the risk of obesity, thus damaging their health.

The article "Impact of the Built Environment on Residents' Health: Evidence from the China Labor Dynamics Survey in 2016" was published in 2023. Journal: J Environ Public Health.

### 4.2. Marginal Effects of the Built Environment on Residents' Health

The meaning of the coefficients estimated based on the ordered probit model is not intuitive and can only be used to identify the direction of the impact of the built environment on residents' health and the significance of the coefficients. Therefore, it is necessary to further calculate the marginal effect of the impact of the built environment on residents' health. The results were shown in Table 3. From the urban scale, the probability of residents' feeling “very healthy” will increase by 31.13% as the urban population density increases by 1 unit, while the probability of feeling “relatively unhealthy” and “ordinary” will decrease by 12.93% and 25.15%, respectively. Every 1-unit increase in road area ratio has the most obvious impact on the “very healthy” level with the probability increasing by 21.68%. On the contrary, the probability of “very unhealthy,” “relatively unhealthy,” and “ordinary healthy” levels will decrease by 1.85%, 9.01%, and 17.52%, respectively. The increase in green area ratio will reduce the probability of “very unhealthy,” “relatively unhealthy,” and “ordinary” levels while improving the probability of “healthy” and “very healthy” levels. Bearing the marginal effect of the urban-built environment variables in mind, the urban population density, road area ratio, and green area ratio are important factors affecting the improvement of residents' health.

In general, the community density has a similar impact on residents' health at all levels, that is, every 1-unit increase in the community population density will lead to a significant increase of the probability of residents' health at “very unhealthy,” “relatively unhealthy,” and “ordinary” levels, and conversely, a decrease at the “healthy” and “very healthy” levels. The results indicate that the higher the community population density, the worse the residents' self-perceived health status. The green coverage ratio only has a significant effect on residents' health at “relatively unhealthy” and “very healthy” levels. Every 1-unit increase in the green coverage ratio will cause a 2.32% decrease in the probability of residents' health at the “relatively unhealthy” level, and conversely, a 5.59% increase at the “very healthy” level.

### 4.3. Robustness Test

To further ensure the rigor of the main conclusions, the following three methods were adopted to conduct the robustness test of Model 4 in Table 2, and the results are shown in Table 4. First, the reliability of the conclusion was further verified by replacing the explained variables. Regarding the residents' health level, as there were only 43 samples at the “very unhealthy” level with a self-perceived health score of 1, accounting for 0.9% of the total samples, therefore, the samples with a self-rated health score of 1 were included in the samples at the “relatively unhealthy” level with a score of 2 for analysis. Second, the selected samples were replaced. According to the limitation of the design of the China Labor Dynamics Survey, in order to reduce the error caused by mixed age, regression analysis was conducted on the adult subsamples as the selected samples included both adults and minors. Finally, the robustness test was carried out using the transformation measurement method. As residents' self-rated health is an ordered discrete variable, the ordered logit model was used in this study to replace the ordered probit model used in benchmark regression for estimation so as to test whether the sign and significance of regression coefficients will be changed.

The article "Impact of the Built Environment on Residents' Health: Evidence from the China Labor Dynamics Survey in 2016" was published in 2023. Journal: J Environ Public Health.

According to the results of the robustness test, the results of test 1 are basically consistent with that of the benchmark regression, while the results of robustness test 2 show that the green space ratio has changed from a significant positive correlation level of 10% to a significant correlation level of 5%. The results of robustness test 3 show that the urban green space ratio and the community green coverage ratio have an insignificant impact on residents' health, and the other conclusions are consistent with the original results. In light of the comprehensive analysis, there is a robust correlation between urban population density, road area ratio, green area ratio, community population density, and green coverage ratio and residents' health, which further confirms the main finding of the benchmark model, that is, the urban- and community-built environment is significantly correlated with residents' health.

### 4.4. Analysis of Age Heterogeneity

Individuals with different characteristics have differentiated perceptions and responses to the built environment; thus, the impact of the built environment on residents' health will also be different. Given that age differences may lead to differences in individual behaviors, preferences, and cognitive levels, it is necessary to further explore whether there is heterogeneity of the built environment on residents' health in different age groups on the basis of the total effect.

To explore age heterogeneity, this study divided the samples into three groups: “samples aged 16–34,” “samples aged 35–55,” and “samples aged over 55.” The regression results are shown in Table 5. Among people aged 16 to 34 years old, the green space ratio at the urban level has no significant impact on their health. The possible reason is that the activity space of this age group is relatively limited, mainly concentrated in schools and at workplace. With limited daytime activities and less exposure to green space, the green availability has less impact on their health, which can also explain that there is an insignificant impact of community population density on their health. Among people aged 35 to 55 years old, the significance and coefficient direction of the impact of the built environment on residents' health at the urban and community scales are basically consistent with the total effect.

The article "Impact of the Built Environment on Residents' Health: Evidence from the China Labor Dynamics Survey in 2016" was published in 2023. Journal: J Environ Public Health.

Among groups aged over 55, bus accessibility at the urban level presents a significantly positive impact on their health. The reason may lie in that people in this age group tend to walk or take a bus rather than driving cars and motorcycles with the decline of their physiological functions. Therefore, preferable bus accessibility can increase the probability of taking a bus trip, thus increasing physical activities and improving their health. Moreover, the impact of the green coverage ratio on this age group changed from a significant positive correlation level of 10% to a significant correlation level of 5%. Compared with young people, people in this age group are more likely to engage in activities in the community and are more sensitive to greenness because of impaired mobility caused by physiological decline and time and space constraints caused by a large number of daily household activities [40]. Besides, older people prefer to do physical exercise in green spaces. A high community green coverage ratio means more types of green space and corresponding facilities, which can boost their physical and mental health by promoting physical activities and social interaction.

### 4.5. Impact Path of the Community Built Environment on Residents' Health

As the most basic part in an urban city, the community is also the fundamental unit for the implementation of the healthy city strategy. However, there is a lack of intensive analysis of the impact pathways of the community-built environment on residents' health in the current research, so further exploration of the action mechanism becomes a necessity. On the basis of Model 2 in Table 2, individual behavioral variables were incorporated in this part to further clarify the impact pattern of the community-built environment on residents' self-rated health through physical exercise, neighborhood support, and community safety.

The article "Impact of the Built Environment on Residents' Health: Evidence from the China Labor Dynamics Survey in 2016" was published in 2023. Journal: J Environ Public Health.

The results in column 2 of Table 6 show the impact of built environment factors on physical exercise at the community scale. Among the built environment factors, there is a significant relationship between community population density, diversity, and green coverage ratio and physical exercise. In terms of population density, the high population density has a greater positive effect on physical exercise and the same as the community diversity. The reason is that the high population density and good diversity shorten the daily travel distance of residents and provide more possibilities for walking trips.

Column 4 in Table 6 reports the impact of built environment factors on neighborhood support. Low community population density helps to promote neighborhood support, and on the contrary, the high population density will weaken the behavior as high-density living space causes an anonymous, indifferent, and lukewarm neighborhood relationship, thus aggravating interpersonal friction [41].

The impact of built environment factors on community safety is presented in Column 6 in Table 6. High population density will reduce the sense of residential security. The possible reason is that most communities in China are relatively weak in cohesion and large heterogeneity of population composition, failing to give full play to the natural monitoring mechanism of “Street Eye” [42]. On the contrary, high density increases the street crime rate [43], thus weakening their sense of residential security. Simultaneously, the green coverage ratio has a significant positive impact on the sense of residential security in communities. Empirical studies on the broken windows theory have shown that the decline of the built environment will increase the crime rate and reduce residents' sense of residential security [44].

Following the bootstrap test, it was found that the mediating effect of physical exercise, neighborhood support, and community safety truly exist. Considering the mediating effect of neighborhood support, the impact pathway of the built environment on residents' health is as follows: the high population density of the community reduces the degree of neighborhood support, which in turn damages residents' health. The impact pathway of community security as the mediating effect is as follows: the increase of community population density causes a weakened perception of residential safety, resulting in the decline of the self-perceived health level, while the green coverage ratio improves residents' health by enhancing their perceived safety.

## 5. Discussion

One of the findings of this study shows that population density exhibits positive and negative effects at the urban and community scales, respectively. On the one hand, a higher level of urban population density will promote residents' health because densely populated cities with a compact spatial structure will reduce travel distances and encourages the nonmotorized travel mode. In addition, according to the research samples, the high-density cities are mainly those with large populations and developed economies where residents often have higher household income and stronger health consciousness, more adequate supply of urban medical resources, and better urban public service; therefore, the urban population density has a positive effect on residents' health from a more macro level. On the other hand, community population density has a negative nonlinear impact on residents; that is, the high community population density will damage residents' physical and mental health. This conclusion runs counter to the urban scale, and as residents usually engage in their daily activities at the workplace and residence, they may be more sensitive to the built environment factors at the community scale. The high-density environment will occupy the public open space, thus limiting the level of the physical activity. In addition, cities with high population density tend to have a faster pace of life, greater psychological pressure, and worse sleep quality, and the crowded environment is likely to lead to a decline in residents' health and comfort. This series of unhealthy lifestyles may be detrimental to their health.

The article "Impact of the Built Environment on Residents' Health: Evidence from the China Labor Dynamics Survey in 2016" was published in 2023. Journal: J Environ Public Health.

Another finding is that there are significant differences in the impact of the built environment on the health of adolescents, young and middle-aged adults, and elderly people, given their markedly different life courses. On the one hand, urban green space only has a positive impact on young and middle-aged adults aged 35–55 but has no impact on the other two age groups. The possible reason is that the other two age groups have more limited activity space, mainly concentrated in schools, workplaces, and near the communities, with limited daytime activities and less touch to green space, so green availability has less impact on their health. Bus accessibility only has a significant positive impact on the middle-aged and elderly population aged 56–64. People at this age prefer to walk and take a bus due to their declined physiological functions. Therefore, better bus accessibility can improve their probability of taking a bus, thus increasing their physical activities and improving their health. On the other hand, community population density has a negative impact on the three age groups; that is, the high community population density will damage their physical and mental health.

The article "Impact of the Built Environment on Residents' Health: Evidence from the China Labor Dynamics Survey in 2016" was published in 2023. Journal: J Environ Public Health.

In addition, this study has also found that the built environment will have an impact on residents' self-rated health via physical activity, neighborhood support, and community safety. According to the impact direction, the compact built environment factors include two categories, namely, the health-promoted built environment factors and the health-damaged built environment factors. The health-promoted built environment factors include higher green coverage ratio. Specifically, higher green coverage ratio can promote residents' self-rated health by improving their perception of residential safety in the community. The health-damaged built environment factors include high community population density. Specifically, high population density not only reduces the degree of neighborhood support but also has a negative impact on the residential safety, thus adversely affecting the residents' health.

## 6. Conclusions

More and more attention has been paid to the studies on the contributory factors of residents' health from the perspective of geography. However, few studies have systematically analyzed the impacts, heterogeneity, and impact mechanisms of various built environment factors from a multiscale perspective. Based on the 4,641 samples in China, this study explored the impact of the built environment on residents' health at the urban and community scales. On the basis of controlling the socio-economic attributes of individuals and households and individual behavior, this study shows that the built environment factors at both the urban and community scales have a significant impact on residents' health, and there are significant differences in this impact among different age groups. This study also reported that the built environment factors at the community level have an impact on residents' health through physical exercise, neighborhood support, and community safety. Furthermore, in this study, population density has different performance on residents' health at different scales. On the one hand, a higher level of urban population density will promote residents' health. On the other hand, community population density has a negative nonlinear effect on residents; that is, high community population density will damage residents' physical and mental health. Therefore, some measures should be taken in the construction of healthy cities. First, it is of necessity to strengthen road connectivity, promote street walkability, and create high-quality street walking space; second, adequate parks and squares should be planned to provide residents with high-quality green space and physical activity space; and third, great efforts should be paid to improve urban functions, optimize resource allocation, maintain a suitable population density in urban community, and promote the healthy development of cities. At the same time, the existence of intermediary paths should be fully considered to maximize the health benefits of the built environment from the supply side. In addition, concerning the difference in the impact of the built environment on residents' health among different age groups, the role of the built environment in promoting residents' health should be maximized, and the negative impact should be minimized when regulating the built environment factors.

The article "Impact of the Built Environment on Residents' Health: Evidence from the China Labor Dynamics Survey in 2016" was published in 2023. Journal: J Environ Public Health.

## Figures and Tables

**Table 1:** Descriptive statistics of the key variables.

Types	Name	Definition	Mean	SD	Min	Max
Explained variable	Self-rated health	Very unhealthy = 1; relatively unhealthy = 2; ordinary = 3; healthy = 4; very healthy = 5	3.763	0.889	1	5

Explanatory variables	Population density	Population density in urban districts (10,000 people/km^2^)	0.125	0.0780	0.006	0.341
	Population size	Total population in urban districts at the end of the year (10,000 people)	379.114	0.0360	28.27	1373.32
	Road area ratio	Road area ratio in urban districts (m^2^)	15.03	6.009	4.370	34.21
	Bus accessibility	Buses ownership per 10,000 people in urban districts (set)	14.75	14.82	1.040	89.34
	Green area ratio	Green area in urban district/total population at the end of the year (m^2^)	49.26	36.69	3.336	191.3
	Land use mixture	Residential land, public facilities, external traffic, municipal public facilities, road square, green space, industrial facilities, storage, and other eight types of land use	0.773	0.0400	0.678	0.876
	Rail traffic	Yes = 1; no = 0	0.485	0.500	0	1
	Community population density					
	0-0.1	(0-0.1] = 1; other = 0	0.141	0.348	0	1
	0.1–0.5	(0.1–0.5] = 1; other = 0	0.199	0.399	0	1
	0.5–1	(0.5–1] = 1; other = 0	0.169	0.375	0	1
	1–1.5	(1–1.5] = 1; other = 0	0.081	0.274	0	1
	1.5–2	(1.5–2] = 1; other = 0	0.086	0.280	0	1
	2–2.5	(2–2.5] = 1; other = 0	0.068	0.251	0	1
	>2.5	(>2.5) = 1; other = 0	0.257	0.437	0	1
	Diversity	Total score of eight types of community public infrastructure and service facilities	4.803	1.527	1	8
	Green coverage ratio	Community green coverage rate (%)	0.412	0.248	0	0.950
	Community pollution	Weighted average value of air pollution, water pollution, soil pollution, and noise pollution	4.613	0.859	1	5

Control variables	Gender	Male = 0; female = 1	0.551	0.497	0	1
	Age	Numerical continuous variable	42.93	13.27	16	64
	Marital status	Married = 1; other = 0	0.782	0.413	0	1
	Social insurance participation	Yes = 1; no = 0	0.890	0.313	0	1
	Highest degree	Illiterate = 0; primary school/private school = 1; junior high school = 2; technical secondary school/vocational high school/general high school = 3; junior college = 4; bachelor's degree = 5; master's degree and above = 6	2.940	1.376	0	6
	Household income per capita	Total household income/family members (Yuan)	33806	424451	0	28800000
	History of smoking	Yes = 0; no = 1	0.754	0.431	0	1
	History of alcohol intake	Yes = 0; no = 1	0.804	0.397	0	1
	Car ownership	Yes = 0; no = 1	0.665	0.472	0	1
	Motorcycle ownership	Yes = 0; no = 1	0.616	0.486	0	1

Mediating variables	Physical exercise	No exercise = 1; 3 times a week and more than 30 minutes = 3; other = 2	1.533	0.540	1	3
	Neighborhood support	Very little = 1; less = 2; ordinary = 3; quite many = 4; a great many = 5	2.940	1.013	1	5
	Community safety	Very unsafe = 1, not very safe = 2, relatively safe = 3, very safe = 4	3.007	0.630	1	4

The article "Impact of the Built Environment on Residents' Health: Evidence from the China Labor Dynamics Survey in 2016" was published in 2023. Journal: J Environ Public Health.

**Table 2:** Overall effects of the built environment on residents' health.

Variables	Model 1	Model 2	Model 3	Model 4
Urban population density	1.0208^*∗∗*^ (0.4237)		1.1341^*∗∗*^ (0.4182)	1.1773^*∗∗*^ (0.4256)
Urban scale	0.0001 (0.0001)		0.0001 (0.0001)	0.0001 (0.0001)
Road area ratio	0.0310^*∗∗∗*^ (0.0056)		0.0340^*∗∗∗*^ (0.0069)	0.0345^*∗∗∗*^ (0.0069)
Bus accessibility	0.0029 (0.0025)		0.0023 (0.0019)	0.0018 (0.0018)
Green coverage ratio	0.0012^*∗*^ (0.0007)		0.0012^*∗*^ (0.0007)	0.0013^*∗*^ (0.0007)
Land use mixture	0.7730 (0.7891)		0.6119 (0.7780)	0.4595 (0.7828)
Rail traffic	−0.0221 (0.1115)		−0.0735 (0.1007)	−0.0783 (0.0980)
Community population density				
0–0.1		−0.1019 (0.1143)	−0.3132^*∗∗∗*^ (0.0973)	−0.3001^*∗∗*^ (0.0983)
0.1–0.5		−0.1002 (0.0953)	−0.1850^*∗*^ (0.1040)	−0.1815^*∗*^ (0.1026)
0.5–1		−0.2157^*∗∗*^ (0.1069)	−0.2428^*∗∗*^ (0.1015)	−0.2305^*∗∗*^ (0.1012)
1–1.5		−0.0329 (0.1702)	−0.1298 (0.1463)	−0.1264 (0.1475)
1.5–2		−0.1974^*∗∗*^ (0.0985)	−0.2256^*∗∗*^ (0.1017)	−0.2217^*∗∗*^ (0.1021)
2–2.5		−0.1845^*∗*^ (0.1061)	−0.2417^*∗∗*^ (0.0973)	−0.2630^*∗∗*^ (0.0967)
>2.5				
Diversity		−0.0289 (0.0237)	−0.0194 (0.0209)	−0.0194 (0.0204)
Green coverage ratio		0.2577^*∗*^ (0.1394)	0.2324^*∗*^ (0.1279)	0.2113^*∗*^ (0.1284)
Environmental pollution		−0.0258 (0.0334)	−0.0094 (0.0318)	−0.0055 (0.0327)
Gender	−0.0488 (0.0309)	−0.0396 (0.0312)	−0.0477 (0.0314)	−0.0440 (0.0402)
Age	−0.0517^*∗∗∗*^ (0.0101)	−0.0523^*∗∗∗*^	−0.0525^*∗∗∗*^ (0.0102)	−0.0525^*∗∗∗*^ (0.0102)
		(0.0104)		
Age square	0.0003^*∗∗*^ (0.0001)	0.0003^*∗∗*^ (0.0001)	0.0003^*∗∗*^ (0.0001)	0.0003^*∗∗*^ (0.0001)
Marital status	0.2613^*∗∗∗*^ (0.0567)	0.2921^*∗∗∗*^ (0.0577)	0.2737^*∗∗∗*^ (0.0573)	0.2518^*∗∗∗*^ (0.0571)
Social insurance participation	−0.1202^*∗*^ (0.0720)	−0.1134 (0.0695)	−0.1021 (0.0691)	−0.1085 (0.0690)
Highest degree	0.0790^*∗∗∗*^ (0.0154)	0.0709^*∗∗∗*^ (0.0159)	0.0752^*∗∗∗*^ (0.0149)	0.0639^*∗∗∗*^ (0.0144)
Household income per capita	4.04 × 10^−8^^*∗∗∗*^ (1.17 × 10^−8^)	3.51 × 10^−8^^*∗∗*^ (1.15 × 10^−8^)	3.95 × 10^−8^^*∗∗∗*^ (1.15 × 10^−8^)	3.89 × 10^−8^^*∗∗∗*^ (9.40 × 10^−9^)
History of smoking				0.0057 (0.0507)
History of alcohol intake				−0.0354 (0.0457)
Car ownership				−0.1336^*∗∗∗*^ (0.0404)
Motorcycle ownership				0.0604 (0.0453)
*N*	4641	4641	4641	4641
Pseudolikelihood	−5614.798	−5647.9803	−5595.2479	−5586.2991

Note. ^*∗∗∗*^, ^*∗∗*^, and ^*∗*^show the test conducted at the significance level of 1%, 5%, and 10%, respectively, and in brackets is the clustering robust standard error.

The article "Impact of the Built Environment on Residents' Health: Evidence from the China Labor Dynamics Survey in 2016" was published in 2023. Journal: J Environ Public Health.

**Table 3:** Marginal effects of the key built environment factors on residents' health.

Variables	Very unhealthy	Relatively unhealthy	Ordinary	Healthy	Very healthy
Urban population density	−0.0265^*∗∗*^ (0.0103)	−0.1293^*∗∗*^ (0.0481)	−0.2515^*∗∗*^ (0.0899)	0.0961^*∗∗*^ (0.0361)	0.3113^*∗∗*^ (0.1130)
Urban scale	−1.85 × 10^−6^ (2.67*e* × 10^−6^)	−9.01 × 10^−6^ (1.3 × 10^−5^)	−1.752 × 10^−5^ (2.51 × 10^−5^)	6.7 × 10^−6^ (9.69 × 10^−6^)	2.168 × 10^−5^ (3.11*e* × 10^−5^)
Road area ratio	−0.0008^*∗∗∗*^ (0.0002)	−0.0038^*∗∗∗*^ (0.0008)	−0.0074^*∗∗∗*^ (0.0014)	0.0028^*∗∗∗*^ (0.0006)	0.0091^*∗∗∗*^ (0.0018)
Bus accessibility	−3.97 × 10^−5^ (4.17 × 10^−5^)	−0.0002 (0.0002)	−0.0004 (0.0004)	0.0001 (0.0002)	0.0005 (0.0005)
Green coverage ratio	−2.94 × 10^−5^^*∗*^ (1.64 × 10^−5^)	−0.0001^*∗*^ (7.66 × 10^−5^)	−0.0003^*∗*^ (0.0001)	0.0001^*∗*^ (0.0001)	0.0003^*∗*^ (0.0002)
Land use mixture	−0.0104 (0.0178)	−0.0505 (0.0866)	−0.0982 (0.1667)	0.0375 (0.0648)	0.1215 (0.2063)
Rail traffic	0.0018 (0.0022)	0.0086 (0.0108)	0.0167 (0.0208)	−0.0064 (0.0080)	−0.0207 (0.0260)
Community population density					
0–0.1	0.0068^*∗∗*^ (0.0025)	0.0330^*∗∗*^ (0.0112)	0.0641^*∗∗*^ (0.0205)	−0.0245^*∗∗*^ (0.0080)	−0.0793^*∗∗*^ (0.0263)
0.1–0.5	0.0041^*∗*^ (0.0024)	0.0199^*∗*^ (0.0114)	0.0388^*∗*^ (0.0218)	−0.0148^*∗*^ (0.0088)	−0.0480^*∗*^ (0.0269)
0.5–1	0.0052^*∗∗*^ (0.0024)	0.0253^*∗∗*^ (0.0114)	0.0492^*∗∗*^ (0.0215)	−0.0188^*∗∗*^ (0.0089)	−0.0609^*∗∗*^ (0.0266)
1–1.5	0.0028 (0.0034)	0.0139 (0.0163)	0.0270 (0.0315)	−0.0103 (0.0124)	−0.0334 (0.0388)
1.5–2	0.0050^*∗∗*^ (0.0024)	0.0244^*∗∗*^ (0.0113)	0.0474^*∗∗*^ (0.0218)	−0.0181^*∗∗*^ (0.0086)	−0.0586^*∗∗*^ (0.0270)
2–2.5	0.0059^*∗∗*^ (0.0023)	0.0289^*∗∗*^ (0.0108)	0.0562^*∗∗*^ (0.0206)	−0.0215^*∗∗*^ (0.0079)	−0.0695^*∗∗*^ (0.0260)
>2.5					
Diversity	0.0004 (0.0005)	0.0021 (0.0022)	0.0041 (0.0044)	−0.0016 (0.0016)	−0.0051 (0.0054)
Green coverage ratio	−0.0048 (0.0030)	−0.0232^*∗*^ (0.0140)	−0.0451 (0.0277)	0.0173 (0.0110)	0.0559^*∗*^ (0.0337
Environmental pollution	0.0001 (0.0007)	0.0006 (0.0036)	0.0012 (0.0070)	−0.0005 (0.0027)	−0.0015 (0.0086)

Note. ^*∗∗∗*^, ^*∗∗*^, and ^*∗*^show the test conducted at the significance level of 1%, 5%, and 10%, respectively.

The article "Impact of the Built Environment on Residents' Health: Evidence from the China Labor Dynamics Survey in 2016" was published in 2023. Journal: J Environ Public Health.

**Table 4:** Robustness test.

Variables	Robustness test 1	Robustness test 2	Robustness test 3
	Replacement of explanatory variables	Adult subsample	Ordered logit model
Urban population density	1.1903^*∗∗*^ (0.4291)	1.1897^*∗∗*^ (0.4231)	1.9980^*∗∗*^ (0.7500)
Urban scale	7.807 × 10^−5^ (0.0001)	7.604 × 10^−5^ (0.0001)	0.0001 (0.0002)
Road area ratio	0.0344^*∗∗∗*^ (0.0069)	0.0344^*∗∗∗*^ (0.0068)	0.0596^*∗∗∗*^ (0.0121)
Bus accessibility	0.0018 (0.0019)	0.0019 (0.0019)	0.0035 (0.0018)
Green space ratio	0.0012^*∗*^ (0.0007)	0.0015^*∗∗*^ (0.0007)	0.0019 (0.0012)
Land use mixture	0.4515 (0.7833)	0.4003 (0.7921)	0.7400 (1.3702)
Rail traffic	−0.0749 (0.0985)	−0.0759 (0.0982)	−0.1307 (0.1704)
Community population density			
0–0.1	−0.2972^*∗∗*^ (0.0999)	−0.2958^*∗∗*^ (0.0984)	−0.4880^*∗∗*^ (0.1720)
0.1–0.5	−0.1787^*∗*^ (0.1035)	−0.1882^*∗*^ (0.1025)	−0.2920 (0.1829)
0.5–1	−0.2265^*∗∗*^ (0.1016)	−0.2412^*∗∗*^ (0.1033)	−0.3911^*∗∗*^ (0.1826)
1–1.5	−0.1142 (0.1461)	−0.1378 (0.1466)	−0.1941 (0.2612)
1.5–2	−0.2222^*∗∗*^ (0.1024)	−0.2060^*∗∗*^ (0.1005)	−0.4035^*∗∗*^ (0.1749)
2–2.5	−0.2666^*∗∗*^ (0.0993)	−0.2779^*∗∗*^ (0.0971)	−0.4510^*∗∗*^ (0.1816)
>2.5			
Diversity	−0.0177 (0.0204)	−0.0171 (0.0207)	−0.0237 (0.0351)
Green coverage ratio	0.2071^*∗*^ (0.1315)	0.2229^*∗*^ (0.1302)	0.3150 (0.2306)
Environmental pollution	−0.0047 (0.0331)	−0.0031 (0.0332)	−0.0092 (0.0591)
Control variable	Controlled	Controlled	Controlled
*N*	4641	4519	4641
Pseudolikelihood	−5455.6575	−5464.052	−5588.9023

Note. ^*∗∗∗*^, ^*∗∗*^, and ^*∗*^show the test conducted at the significance level of 1%, 5%, and 10%, respectively, and in brackets is the clustering robust standard error.

**Table 5:** Age heterogeneity.

Variables	Samples aged 16–34	Samples aged 35–55	Samples aged over 55
Urban population density	0.6835 (0.6325)	1.3626^*∗∗*^ (0.4819)	1.4857^*∗∗*^ (0.5671)
Urban scale	−2.955 × 10^−5^ (0.0002)	0.0002 (0.0001)	5.81 × 10^−6^ (0.0002)
Road area ratio	0.0384^*∗∗∗*^ (0.0099)	0.0344^*∗∗∗*^ (0.0080)	0.0315^*∗∗∗*^ (0.0085)
Bus accessibility	0.0016 (0.0020)	0.0014 (0.0023)	0.0182^*∗∗∗*^ (0.0057)
Green space ratio	−8.95 × 10^−6^ (0.0009)	0.0021^*∗∗*^ (0.0008)	0.0009 (0.0011)
Land use mixture	1.3273 (1.0316)	0.1861 (0.9354)	0.0131 (1.1541)
Rail traffic	0.0430 (0.1348)	−0.1751 (0.1069)	−0.1076 (0.1367)
Community population density			
0–0.1	−0.2817^*∗*^ (0.1521)	−0.3389^*∗∗*^ (0.1184)	−0.2126 (0.1640)
0.1–0.5	−0.0255 (0.1366)	−0.1891^*∗*^ (0.1107)	−0.3485^*∗∗*^ (0.1497)
0.5–1	−0.0417 (0.1475)	−0.2627^*∗∗*^ (0.1245)	−0.4178^*∗∗∗*^ (0.1252)
1–1.5	−0.1144 (0.2343)	−0.1016 (0.1571)	−0.2276 (0.1668)
1.5–2	−0.2447^*∗*^ (0.1369)	−0.2229^*∗∗*^ (0.1089)	−0.1783 (0.1396)
2–2.5	−0.0819 (0.1570)	−0.3497^*∗∗*^ (0.1274)	−0.3102^*∗∗*^ (0.1029)
>2.5			
Diversity	0.0096 (0.0292)	−0.0317 (0.0247)	−0.0345 (0.0245)
Green coverage ratio	0.1182 (0.1818)	0.1804 (0.1449)	0.4249^*∗∗*^ (0.1593)
Environmental pollution	−0.0028 (0.0483)	0.0047 (0.0368)	−0.0171 (0.0567)
Control variable	Controlled	Controlled	Controlled
*N*	1371	2381	889
Pseudolikelihood	−1444.4917	−2968.4793	−1120.4991

Note. ^*∗∗∗*^, ^*∗∗*^, and ^*∗*^show the test conducted at the significance level of 1%, 5%, and 10%, respectively, and in brackets is the clustering robust standard error.

The article "Impact of the Built Environment on Residents' Health: Evidence from the China Labor Dynamics Survey in 2016" was published in 2023. Journal: J Environ Public Health.

**Table 6:** Regression results of the community-built environment, mediating variables, and residents' health.

Variables	Self-rated health	Mediating variable 1		Mediating variable 2		Mediating variable 3	
		Physical exercise	Self-rated health	Neighborhood support	Self-rated health	Community safety	Self-rated health
Physical exercise			0.0891^*∗∗*^ (0.0391)				
Neighborhood support					0.1173^*∗∗∗*^ (0.0206)		
Community safety							0.2407^*∗∗∗*^ (0.0309)
Community population density							
0-0.1	−0.0820 (0.1165)	0.1005 (0.1241)	−0.0855 (0.1161)	0.3406^*∗∗*^ (0.1546)	−0.1192 (0.1211)	−0.0315 (0.1394)	−0.0774 (0.1141)
0.1–0.5	−0.0892 (0.0945)	0.0943 (0.1024)	−0.0927 (0.0946)	0.1364 (0.1050)	−0.1057 (0.0967)	0.0868 (0.1186)	−0.1005 (0.0923)
0.5–1	−0.2016^*∗*^ (0.1065)	−0.0271 (0.1058)	−0.2007^*∗*^ (0.1077)	−0.0193 (0.0925)	−0.2012^*∗*^ (0.1088)	−0.1601 (0.1417)	−0.1821^*∗*^ (0.1063)
1–1.5	−0.0281 (0.1726)	0.2816^*∗∗*^ (0.1084)	−0.0384 (0.1703)	0.0047 (0.1490)	−0.0280 (0.1673)	−0.2550^*∗*^ (0.1519)	0.0081 (0.1630)
1.5–2	−0.1990^*∗*^ (0.1017)	0.1691 (0.1164)	−0.2055^*∗∗*^ (0.0993)	−0.2035^*∗*^ (0.1060)	−0.1771^*∗*^ (0.1011)	−0.0417 (0.1166)	−0.1962^*∗*^ (0.1037)
2–2.5	−0.1949^*∗*^ (0.1045)	0.2959^*∗∗*^ (0.0997)	−0.2067^*∗*^ (0.1058)	0.0111 (0.1869)	−0.1975^*∗∗*^ (0.1000)	−0.2740^*∗*^ (0.1614)	−0.1595 (0.0997)
>2.5							
Diversity	−0.0298 (0.0233)	0.0428^*∗*^ (0.0232)	−0.0314 (0.0233)	−0.0027 (0.0243)	−0.0297 (0.0232)	−0.0007 (0.0248)	−0.0301 (0.0226)
Green coverage ratio	0.2365^*∗*^ (0.1389)	−0.1111 (0.1493)	0.2266^*∗*^ (0.1398)	0.2146 (0.1723)	0.2156 (0.1401)	0.6426^*∗∗∗*^ (0.2106)	0.1566 (0.1335)
Environmental pollution	−0.0246 (0.0338)	0.0183 (0.0427)	−0.0252 (0.0340)	−0.0066 (0.0362)	−0.0243 (0.0331)	−0.0319 (0.0547)	−0.0209 (0.0324)
Socio-economic attributes	Controlled	Controlled	Controlled	Controlled	Controlled	Controlled	Controlled
Individual behavior variable	Controlled	Controlled	Controlled	Controlled	Controlled	Controlled	Controlled

Note. ^*∗∗∗*^, ^*∗∗*^, and ^*∗*^show the test conducted at the significance level of 1%, 5%, and 10%, respectively, and in brackets is the clustering robust standard error.

The article "Impact of the Built Environment on Residents' Health: Evidence from the China Labor Dynamics Survey in 2016" was published in 2023. Journal: J Environ Public Health.

## Data Availability

The data can be made available on a reasonable request by contacting the corresponding author.
